# Synthesis, Characterization, Antimicrobial Studies and Corrosion Inhibition Potential of 1,8-dimethyl-1,3,6,8,10,13-hexaazacyclotetradecane: Experimental and Quantum Chemical Studies

**DOI:** 10.3390/ma9020107

**Published:** 2016-02-11

**Authors:** Henry U. Nwankwo, Collins N. Ateba, Lukman O. Olasunkanmi, Abolanle S. Adekunle, David A. Isabirye, Damian C. Onwudiwe, Eno E. Ebenso

**Affiliations:** 1 Department of Chemistry, School of Mathematical & Physical Sciences, Faculty of Agriculture, Science and Technology, North-West University (Mafikeng Campus), Private Bag X2046, Mmabatho 2735, South Africa; henrynwankwo16@gmail.com (H.U.N.); waleolasunkanmi@gmail.com (L.O.O.); sadekpreto@gmail.com (A.S.A.); David.Isabirye@nwu.ac.za (D.A.I.); dcconwudiwe@gmail.com (D.C.O.); 2 Material Science Innovation & Modelling (MaSIM) Research Focus Area, Faculty of Agriculture, Science and Technology, North-West University (Mafikeng Campus), Private Bag X2046, Mmabatho 2735, South Africa; 3 Department of Microbiology, School of Environmental and Health Sciences, Faculty of Agriculture, Science and Technology, North-West University (Mafikeng Campus), Private Bag X2046, Mmabatho 2735, South Africa; 16528026@nwu.ac.za; 4 Department of Chemistry, Faculty of Science, Obafemi Awolowo University, Ile-Ife 220005, Nigeria

**Keywords:** macrocycles, dematallation, antimicrobial, anticorrosion, electrochemical, NBO analysis, J0101

## Abstract

The macrocylic ligand, 1,8-dimethyl-1,3,6,8,10,13-hexaazacyclotetradecane (MHACD) was synthesized by the demetallation of its freshly synthesized Ni(II) complex (NiMHACD). Successful synthesis of NiMHACD and the free ligand (MHACD) was confirmed by various characterization techniques, including Fourier transform infra-red (FT-IR), proton nuclear magnetic resonance (^1^H-NMR), carbon-13 nuclear magnetic resonance (^13^C-NMR), ultraviolet-visible (UV-vis), and energy dispersive X-ray (EDX) spectroscopic techniques. The anti-bacteria activities of MHACD were investigated against *Staphylococcus aureus* and *Enterococcus* species and the results showed that MHACD possesses a spectrum of activity against the two bacteria. The electrochemical cyclic voltammetry study on MHACD revealed that it is a redox active compound with promising catalytic properties in electrochemical applications. The inhibition potential of MHACD for mild steel corrosion in 1 M HCl was investigated using potentiodynamic polarization method. The results showed that MHACD inhibits steel corrosion as a mixed-type inhibitor, and the inhibition efficiency increases with increasing concentration of MHACD. The adsorption of MHACD obeys the Langmuir adsorption isotherm; it is spontaneous and involves competitive physisorption and chemisorption mechanisms. Quantum chemical calculations revealed that the energy of the highest occupied molecular orbital (HOMO) of MHACD is high enough to favor forward donation of charges to the metal during adsorption and corrosion inhibition. Natural bond orbital (NBO) analysis revealed the presence of various orbitals in the MHACD that are capable of donating or accepting electrons under favorable conditions.

## 1. Introduction

Macrocyclic ligands are important class of organic compounds that usually contain heteroatoms that are capable of chelating with substrates in their molecules [1]. Most macrocyclic ligands contain nine or more atoms including at least three electron pair donors in their rings [2]. These compounds have received reasonable attention for many years owing to some unique properties that are attributed to the macrocyclic environment present in their molecular structures. Among their distinct characteristics are high thermodynamic stability, the ability of the central metal to exist in unusual oxidation states and their ability to mimic the structural and functional characteristics of naturally occurring macrocyclic molecules [3,4]. These compounds have been reported to have potential applications in biological systems, magnetochemistry, medicine, technology, chemical sensors, precursors to new conducting materials, ladder polymers, dyes and also as catalysts [4,5,6]. Many nitrogen containing macrocyclic compounds are found as fragments of many natural products, fine chemicals and several biologically active compounds [7]. Various nitrogen-containing macrocyclic ligands have been reportedly used as antifungal [8,9,10,11], antibacterial [5,10,11], hypolipidemic [12], anticancer [13], antihistaminic [14], analgesic [15,16], antitubercular [17,18], anticonvulsant [19], anti-inflammatory [15,16,20] anti-tumor [8] and anti-HIV agents [21]. Their potential applications as corrosion inhibitors cannot be ruled out because compounds with N, S, O and P heteroatoms are generally known to possess anticorrosion properties and the corrosion inhibition potentials of a number of macrocycles have been reported [22,23,24,25,26,27].

Fully saturated macrocyclic complexes consisting of six nitrogen atoms such as 1,8-dimethyl-1,3,6,8,10,13-hexaazacyclotetradecane are considerably less common [28,29]. The three general methods of preparing macrocyclic compounds as discussed by Melson [30] include metal template synthesis, complexation method and synthesis involving modification of the macrocyclic ligand and/or the metal ion complex. However, previous attempts to separate 1,8-dimethyl-1,3,6,8,10,13-hexaazacyclotetradecane (MHACD) ligand from its nickel complexes by treating the complexes with excess sodium cyanide, hydrogen sulfide gas, or strong acid had been unsuccessful [29]. The metal complex is identified with an enhanced stability due to a more favorable enthalpy. This is also related to the decreased ligand solvation of the macrocycle, which has less H-bonded water to be displaced in the complex-formation process [31]. This has made it rather impossible to study the antimicrobial and other prospective properties of the metal-free macrocylic ligand MHACD.

This has motivated us to carry out the present study on the synthesis of MHACD via dematallation of its nickel(II) complex (NiMHACD). Successful demetallation was confirmed by various characterization methods including Fourier transform infrared (FT-IR) spectroscopy, nuclear magnetic resonance (NMR) spectroscopy, ultraviolet-visible (UV-vis) adsorption spectroscopy, and energy dispersion X-ray (EDX) techniques. In view of diverse applications of nitrogen-containing macrocyclic ligands as documented in literature [5,6,7,8,9,10,11,12,13,14,15,16,17,18,19,20,21,22,23,24,25,26,27], the present work also investigates some potential applications of MHACD. These include its antimicrobial actions, electrochemical redox activities and corrosion inhibition properties. The antimicrobial properties of MHACD were investigated on *Staphylococcus aureus* and *Enterococcus* species, while the anticorrosion potential was carried out on mild steel in 1 M HCl solution. The choice of 1 M HCl as the test solution for the corrosion inhibition study is premised on the frequent use of dilute hydrochloric acid in various industrial applications [22]. It constitutes a strong corrosive medium and possesses imminent threat to the lifespan of steel materials and other metal-based gadgets. Quantum chemical calculations including the natural bond orbital (NBO) analysis of MHACD are also reported. To the best of our knowledge, this is the first time a study involving these details is being reported on MHACD.

## 2. Results and Discussion

### 2.1. Synthesis and Characterization of NiMHACD and MHACD

The synthesis and characterization of NiMHACD and MHACD are summarized under the experimental section. The spectroscopic data to support successful synthesis of both NiMHACD and MHACD are listed in Table 1. Successful synthesis of NiMHACD was confirmed by the presence of relevant peaks in the FT-IR spectra (Table 1) including the band at 1503 cm^−1^ for N–H bending vibrations, the broad band at 3550 cm^−1^ for N–H stretching and the band at the C–N band at 1026 cm^−1^. The ^13^C-NMR spectra (Table 1) shows three peaks corresponding to the presence of three different chemical environments for the carbon atoms, which is in accordance with the molecular structure of NiMHACD. The peaks at 39.90 and 71.20 ppm for –N–CH_3_ and –N–C–N– respectively are in good agreement with what had been reported in the literature [29]. The ^1^H-NMR spectra (Table 1) gave well-resolved peaks that matched with the structure of the complex. The EDX spectra (Table 1) showed up to 22.5 % Ni confirming the presence of Ni in the NiMHACD. The electronic absorption bands of NiMHACD shown in Figure 1 (also in Table 1) revealed UV-vis absorptions at 324 and 214 nm corresponding to ^1^A_1g_ → ^1^B_1g_ and ^1^A_1g_ → ^1^A_2g_ transitions, respectively, suggesting that NiMHACD is a square planar complex. These bands are in agreement with literature values for square planar configuration around Ni(II) ion in a similar complex [32].

Successful removal of the central Ni from NiMHACD was verified by the relative shifts in the FTIR bands (Table 1) of the isolated ligand, MHACD, compared to the spectra of NiMHACD. The N–H stretching band in MHACD is broader and shifted by about 250 cm^−1^ compared to that of NiMHACD by appearing at 3300 cm^−1^. The ^13^C-NMR of MHACD (Table 1) also showed three distinct chemical environments for carbon atoms with obvious shifts in the peak positions compared to the NiMHACD. There is no significant difference in the ^1^H-NMR data of NiMHACD and MHACD. The UV-vis absorption spectra of MHACD (Figure 1 and Table 1) showed a single peak at 268 nm, which can be assigned to n → σ* transition, while the EDX spectra did not show any peak for the Ni. These observations suggest successful removal of Ni from MHACD to produce the free ligand, MHACD.

### 2.2. Antimicrobial Study

The MHACD was tested for possible activities against bacteria isolates from milk and groundwater samples. The *Staphylococcus aureus* and *Enterococcus* species isolates from milk and groundwater samples were utilized for the assessment of antibacterial activities of MHACD. The diameters of inhibition zone (mm) and the concentration dependencies of the antibacterial activities of MHACD are shown in Figure 2.

The results showed that MHACD has a spectrum of activities against the selected microbes being more active against the *Enterococcus* species and the strength of antimicrobial activities generally increases with increasing concentration from 1 µg/mL to 4 µg/mL. The observed antimicrobial properties of MHACD may be attributed to the presence of N-donor groups in the molecule, which may serve as binding sites to favor the possible binding mechanism that leads to the deactivation of the microbes.

### 2.3. Electrochemical Behavior of MHACD: Cyclic Voltammetry Study

The cyclic voltammogramms (CVs) obtained for Pt electrode in the phosphate buffer solution (PBS) at the scan rate (ν) of 25 mV·s^−1^ without and with 1 mM of MHACD are shown in Figure 3. The effect of scan rate, ν (25 to 300 mV·s^−1^) on the electrochemical behavior of MHACD was also investigated and reported in Figure 4. The CV showed a well-defined redox peaks at positions (I) and (II) (Figure 3a), which can be attributed to the ring redox process. The redox reversible process at 0.3 V indicates that the ring of the synthesized ligand MHACD is electroactive. Similar redox peaks have been reported by Postlethwaite *et al*. [33] for thiol-derivatized porphyrins, which is also a macrocycle. Another anodic peak observed around 1.3 V in the PBS solution containing 1 mM of MHACD (I) (Figure 3b), which was not observed in the blank PBS (Figure 3b) was attributed to the oxidation process of MHACD suggesting that it is electroactive and may function as a catalyst in some electrochemical applications such as chemical and biochemical sensors, fuel cells, *etc*.

The effect of scan rate on the electrocatalytic oxidation of MHACD at the Pt electrode as reported in Figure 4 revealed that the oxidation peak shifted to more positive potentials with increasing scan rate which confirms diffusion kinetic limitation in the electrochemical reaction. It can be observed that when ν > 0.02 *Dcc*, the anodic peak potential, E_pa_ was significantly linearly dependent on the log ν giving rise to the regression equation:

(1) $$E_{pa}=0.0213\log\upsilon +0.122\;(R^{2}=0.9907)$$

The plots of log I_p_ (peak current) *versus* log ν and E_p_ *versus* log ν are shown in Figure 5. As shown in Figure 5a, the current is greatly enhanced with increasing scan rate. Furthermore, the plots of log I_p_ *vs.* log ν (Figure 5a) and E_p_ *vs.* log ν (Figure 5b) exhibit linear behaviors with slight deviation from zero intercept characteristic of a true diffusion process [34,35]. This suggests that there is interplay of electrochemical and chemical processes at the electrode surface. As shown in Equation (1), the Tafel equation for a totally irreversible diffusion-controlled process [36] gave a slope of 0.0213 V·dec^−1^ corresponding to a Tafel value of 42.6 mV·dec^−1^, which is lower than the theoretical value of 118 mV·dec^−1^ often associated with the presence of a one-electron process in the rate-determining step. This suggests the occurrence of either adsorption or involvement of reaction intermediates on the electrode surface [37,38]. The results therefore suggest the possibility of oxidation or chelation of the highly lipophilic ligand, MHACD, on the surface of the Pt electrode as indicated by the oxidation peak at around 1.3 V.

### 2.4. Corrosion Inhibition Study

#### 2.4.1. Potentiodynamic Polarization Measurements

The Potentiodynamic polarization curves for MS in 1 M HCl without and with various concentrations of MHACD are shown in Figure 6. It is apparent from Figure 6 that the polarization curves shifted to lower current regions in the presence of the inhibitor compared to the blank acid medium. This suggests that the synthesized ligand, MHACD, reduces the corrosion current density, which is an indication of its corrosion inhibition potential. The polarization curve in the presence of 10 ppm MHACD appears at relatively more cathodic potential compared to the blank, while the curves appear at relatively more anodic potentials at higher concentrations of MHACD. This suggests that the inhibitive effect of MHACD is more cathodic at 10 ppm than at higher concentrations. The electrochemical kinetic parameters obtained from the Tafel extrapolations are listed in Table 2. It is evident from the results that the maximum shift in the E_corr_ in the presence of the inhibitor relative to the blank acid is 31 mV observed at 10 and 1000 ppm of MHACD. An inhibitor can be classified as a cathodic or anodic inhibitor only if the displacement in E_corr_ is greater than 85 mV; otherwise, it is a mixed-type inhibitor [26,27,39,40,41,42,43,44,45,46]. The slight shift in E_corr_ in the present study implies that the studied inhibitor is a mixed-type inhibitor, which means that the synthesized ligand, MHACD, retards both the anodic dissolution of MS in HCl and the cathodic hydrogen ion reduction process. The values of the Tafel slopes *b*_a_ and *b*_c_ changed with change in concentration of the inhibitor. This suggests that the rate of the corrosion reaction of MS in the acid is affected by the change in concentration of the inhibitor.

The *b_c_* values are generally higher than the *b_a_* values and the change in the Tafel slopes in the presence of the inhibitor relative to the blank acid system is generally higher for the *b_c_*. This observation suggests that the inhibitive effect of MHACD is more pronounced on cathodic hydrogen gas evolution than anodic MS dissolution reaction [45]. In other words, MHACD is a mixed-type inhibitor with predominantly cathodic inhibitive effects. The corrosion current density (*i_corr_*) decreases with increasing concentration of the inhibitor, which is also an indication of the inhibitive effect of MHACD. The values of the percentage inhibition efficiency (%IE_PDP_) also revealed that the inhibition efficiency increases with increasing concentration.

#### 2.4.2. Adsorption Isotherm

The inhibition of metal corrosion by organic molecules is usually as a result of adsorption of the inhibitor molecules on the metal surface. Therefore, an insight into the inhibition mechanism can be gained from the adsorption isotherm. The adsorption of an organic adsorbate onto metal–solution interface can be represented by a substitutional adsorption process between the organic molecules in the aqueous solution phase (Org_(sol)_) and the water molecules on the metallic surface (H_2_O_(ads)_) according to the equation:

(2) Org_(sol)_ + *x* H_2_O_(ads)__⇌_ Org_(ads)_ + *x* H_2_O_(sol)_

where *x* is the size ratio of the number of water molecules replaced by one molecule of organic substrate. Adsorption isotherms are often employed to gain more insights into the mechanism of corrosion inhibition, due to the fact that thermodynamic adsorption parameters provide information about the mode of interactions between the inhibitor molecules and the active sites on the metal surface [47,48,49,50,51]. The experimental data in the present study were subjected to various adsorption isotherms including Langmuir, Temkin, Freundlich, Frumkin and Flory–Huggins but the Langmuir adsorption isotherm gave the best correlation. Therefore, thermodynamic adsorption parameters for MS in 1 M HCl in the presence of the studied inhibitor were obtained from the Langmuir isotherm plot of the form:

(3) $$\frac{C_{\text{inh}}}{\theta }\;=\;\frac{1}{K_{\text{ads}}}\;+\;C_{\text{inh}}$$

where θ is the degree of surface coverage, *K*_ads_ is the equilibrium constant of the adsorption process and *C_inh_* is the concentration of the inhibitor. The Langmuir adsorption isotherm plot is shown in Figure 7, indicating near unity values of slope and correlation coefficient (R^2^). The adsorption equilibrium constant, K_ads_, was obtained from the intercept and the change in Gibb’s free energy (∆G_ads_) for the adsorption process was obtained using the equation:

(4) ∆G°_ads_ = −RT ln (55.5 K_ads_)

where R is the universal gas constant, T is absolute temperature and 55.5 is the molar concentration of water in solution.

Since the K_ads_ represents the degree of adsorption, a high value of *K*_ads_ signifies that the inhibitor is strongly adsorbed on the steel surface [42,48,49,52,53]. The value of 10,660 L/mol obtained for the K_ads_ in the present study is an indication of strong adsorption of the molecules of MHACD to the steel surface.

The value of ΔG_ads_ is often used to classify the adsorption process as physisorption, chemisorption or a combination of both. Generally, a value of ΔG_ads_ around −20 kJ·mol^−1^ or less negative suggests that the adsorption process involves electrostatic interactions between the charged molecules and the charged metal surface, termed physisorption, whereas a value of ΔG_ads_ around −40 kJ·mol^−1^ or more negative indicates the involvement of charge sharing or transfer from organic molecules to the metal surface during the adsorption process leading to the formation of coordinate bond and the adsorption process is termed chemisorption [48,49,50,51,52,53]. The value of 33.48 kJ·mol^−1^ obtained for ∆G_ads_ in the present study lies in-between the thresholds for physisorption and chemisorption mechanisms suggesting that the adsorption of the synthesized ligand on MS surface in 1 M HCl involves competitive physisorption and chemisorption mechanisms [44,45,51].

#### 2.4.3. Quantum Chemical Study

The optimized structure of MHACD is shown alongside the highest occupied molecular orbital (HOMO) and lowest unoccupied molecular orbital (LUMO) electron density surfaces in Figure 8. The optimized geometry parameters of MHACD are listed in Table 3. The values of the bond lengths in the optimized structure of MHACD revealed that most of the atoms that are supposedly in the same chemical environments are not equivalent.

This is reflected in the unequal values of the bond lengths found for bonds like C9–N5 and C35–N30; C6–N12 and C9–N14; *etc*. The bond lengths for the geminal C–H bonds (not shown) are also not equal. This indicates that the molecule is non-symmetric. The observed bond angles and dihedral angles (not shown) also revealed the non-planarity of the molecule. The HOMO graphical surface revealed that the HOMO orbitals are of sigma type as expected for the saturated molecule, and distributed over the C and N atoms in the ring and not extended to the C-atoms C1 and C39 of substituent methyl groups. The LUMO on the other hand is mainly found on the C1 and slightly extended to the vicinal C and N atoms. Some calculated quantum chemical parameters of MHACD are listed in Table 4. Due to the sparseness of reports on the frontier molecular orbital (FMO) energies of similar organic molecules, the E_HOMO_ and E_LUMO_ of the synthesized ligand were compared with our recent reports on some macrocylic compounds such as porphyrins [26], phthalocynanins and naphthalocyanins [27]. The HOMO and the LUMO of the studied ligand are less stable compared to those of porphyrins [26], phthalocynanins and naphthalocyanins [27]. This suggests that the studied ligand may have better electron-donating ability than phthalocynanin and naphthalocyanin. The values of global electronegativity (χ) and hardness (η) of MHACD are also listed in Table 4. The value of ∆N is a gauge of donor–acceptor characteristics of an inhibitor and subsequently its effect on inhibition potential. According to Lukovits *et al*. [54], and as reported in some of our recent studies [27,39,46], a value of ∆N less than 3.6 indicates that the inhibition efficiencies of an inhibitor tend to increase by increasing the electron-donating ability to the metal surface. Negative values of ∆N suggest that the inhibition of metal corrosion is predominately controlled by retro-donation from the metal to the inhibitor molecule [27]. The value of ∆N obtained for the synthesized ligand in the present study is positive and less than 3.6, which suggests that the inhibitive action of the ligand is mainly as a result of forward donation to the appropriate vacant orbitals of the metal and that the inhibition efficiency of MHACD tends to increase with increasing electron-donating ability.

To investigate the prospective orbitals in the molecule of MHACD that can donate and accept charges to/from the appropriate orbital of the metal, a full natural bond orbital (NBO) analysis was carried out. The abridged natural atomic orbital (NAO) occupancies are listed in Table 5. The N atoms being lone-pair carriers were found to have higher occupancies than the C atoms. The results in Table 4 therefore showed only the occupancies of the valence orbitals of the N atoms, while the lowest energy Rydberg orbitals of C and N atoms in the molecule of MHACD are also listed in Table 6. Since the 2p orbital is generally of higher energy than the 2s orbital, the 2p orbital are considered to have better tendency of donating electrons to the appropriate vacant orbital of the metal. The highest energy orbitals in each of the six N atoms contained in the molecule of MHACD, as shown in Table 5, are 2py (N5), 2pz (N12), 2px (N14), 2px (N28), 2px (N30) and 2py (N38), such that the comparative order of increasing energy of the highest energy orbitals in each of the six N atoms is 2px (N30) > 2px (N14) > 2px (N28) > 2pz (N12) > 2py (N38) > 2py (N5). This observation suggests that the N30 atom has the highest tendency to interact with the lowest energy vacant p-orbitals of Fe in favor of forward donation. The possibility of retro-donation cannot be completely ruled out in corrosion inhibition mechanism due to the general complexity of adsorption phenomenon. For this reason, the relative tendencies of the C and N atoms to accept electrons from the occupied d-orbitals of Fe were investigated by considering the relative energies of their Rydberg (3d) orbitals. Rydberg orbitals are not occupied in ground state electronic configurations due to their relatively high energy values. The lower the energy of a Rydberg orbital, the more stable the orbital and the better the tendency of the orbital in accepting electrons from appropriate orbitals of donor specie. The results, as shown in Table 5, revealed that C19 (3dz^2^) has the highest tendency of electron acceptance from the d-orbitals of Fe followed by C25 (3dz^2^), then N38 (3dxz) and N30 (3dz^2^).

## 3. Experimental Section

### 3.1. Materials, Reagents and Strains

All chemicals and reagents were of analytical grade and were used without further purification. Methanol (CH_3_OH), formaldehyde (CH_2_O), ethylenediamine (C_2_H_8_N_2_), methylamine (CH_3_NH_2_), acetonitrile (CH_3_CN), sodium cyanide, sodium hydroxide (NaOH) pellets, hydrochloric (HCl) acid, sodium dihydrogen orthophosphate dihydrate (NaH_2_PO_4_·2H_2_O), disodium hydrogen orthophosphate (Na_2_HPO_4_), potassium ferrocyanide(II) (K_4_Fe(CN)_6_·3H_2_O), potassium hexacyano-ferrate(III) (C_6_FeK_3_N_6_) were commercially obtained from MERCK (Sandton, South Africa) and SIGMA-ALDRICH (Aston Manor, South Africa). Müller-Hinton Agar was purchased from Fluka (New York, NY, USA). Microorganisms (*Staphylococcus aureus* and *Enterococci)* were obtained from the culture collection of the Department of Biological sciences, North-West University (Mafikeng Campus), Mmabatho, South Africa. Analytical reagent grade of disodium hydrogen orthophosphate, potassium ferrocyanide(II) and potassium hexacyano-ferrate(III) were utilized to prepare 0.1 mol·L^−1^ Phosphate buffer solution and 5 mM Fe(CN)_6_^3−/4−^ respectively.

### 3.2. Synthesis

#### 3.2.1. Synthesis of 1,8-dimethyl-1,3,6,8,10,13-hexaazacyclotetradecanenickel(II) Complex (NiMHACD)

The preparation of 1,8-dimethyl-1,3,6,8,10,13-hexaazacyclotetradecanenickel(II) complex (NiMHACD) was carried out as reported in the literature [26]. Nickel (II) chloride hexahydrate (11.5 g), ethylenediamine (6.8 mL), formaldehyde (20 mL), and methylamine (8.6 mL) were slowly added to methanol solution (50 mL) with continuous stirring. The mixture was heated under reflux for 24 h until a dark orange solution was formed. The solution was cooled in an ice-bath, followed by filtration to remove nickel hydroxide. Excess perchloric acid was added to the filtrate and the resulting mixture was kept in an ice-bath for 24 h until the formation yellow crystalline product. The yellow crystals were washed in a mixture of ether and methanol, and then air-dried. The crystals were further recrystallized from boiling water to obtain the final product, (NiMHACD).

FTIR (v/cm^−1^): 1026s (C–N); 1503m (N–H, bend); 3222m (C–H, stretch), 3550b (N–H, stretch) ^13^CNMR (CDCl_3_, δ, ppm ): three distinct peaks: 39.90 (–N–CH_3_), 71.20 (–N–C–N–), 172.60 (–N–CH_2_–CH_2_–N)
^1^HNMR (CDCl_3_, δ, ppm ): 0.9 (s, 6H, –N–CH_3_), 1.2 (m, 8H, –N–CH_2_–CH_2_–N–), 1.5 (d, 8H, –N–CH_2_–N–), 7.2 (m, 4H, –C–NH–C–)
UV-vis (nm): 214 (^1^A_1g_→^1^A_2g_), 324 nm (^1^A_1g_→^1^B_1g_)
EDX: 22.5 % Ni

The synthetic route is summarized in the schematic diagram as shown in Figure 9.

#### 3.2.2. Synthesis of 1,8-dimethyl-1,3,6,8,10,13-hexaazacyclotetradecane (MHACD) by Demetallation of NiMHACD

Aqueous solutions (10 mL each) of the initially synthesized nickel (II) complex, NiL (5.64 g), sodium hydroxide pellets (6 g) and sodium cyanide (10 g) were mixed together and evaporated in a rotary evaporator until excess liquid was removed. The resulting crystalline solid was washed with acetonitrile and excess chloroform, and finally evaporated to dryness. The white crystalline solid was collected and air-dried to obtain MHACD as the final product.

FTIR (v/cm^−1^): 1421s (C–N); 1584m (N–H, bend); 3300b (N–H, stretch)
^13^CNMR (CDCl_3_, δ, ppm): three distinct peaks: 28.56 (–N–CH_3_), 78.43 (–N–C–N–), 174.60 ()
^1^HNMR (CDCl_3_, δ, ppm): 0.9 (s, 6H, –N–CH_3_), 1.3 (m, 8H, –N–CH_2_–CH_2_–N–), 1.6 (d, 8H, –N-CH_2_–N–), 7.3 (m, 4H, –C–NH–C–)
UV-vis (nm): 286 (n→σ*)
EDX: 0 % Ni

The synthetic route of MHACD is summarized in the schematic diagram as shown in Figure 10.

### 3.3. Spectroscopic Analyses

Spectroscopic analyses were carried out on both the synthesized complex, NiMHACD and the free ligand, MHACD. FTIR spectrophotometer (Cary 600 series FTIR spectrophotometer obtained from Agilent Technology, Johannesburg, South Africa) and the UV-vis spectrophotometer (Cary 300 series UV-vis spectrophotometer obtained from Agilent Technology, Johannesburg, South Africa) were used for the FTIR and UV-vis studies respectively. The infrared spectra were recorded between 700 and 4000 cm^−1^ while the UV-vis electronic absorption spectra were recorded in the wavelength range of 200–400 nm. Energy Dispersive X-ray (EDX) spectra were carried out with EDX-720 obtained from Shimadzu (Westville, South Africa). The proton (^1^H) and carbon-13 (^13^C) NMR spectra of the compounds were recorded on a Varian Gemini 300 Broadband NMR spectrometer at 300 MHz in CDCl_3_.

### 3.4. Electrochemical Characterization of MHACD: Cyclic Voltammetry (CV) Study

Electron transport properties of MHACD were investigated by electrochemical experiment using the cyclic voltammetry (CV) technique. The CV profile was recorded for a 10^−3^ M solution of the synthesized ligand prepared in 0.1 M phosphate buffer solution (PBS). A 5 mM Fe(CN)_6_^3−/4−^ solution was used as the redox probe. The effect of scan rates on the electrochemical behavior of MHACD was observed between 25 and 300 mV·s^−1^. Electrochemical studies were carried out on Metrohm Autolab potentiostat/galvanostat PGSTAT 302N supplied by Eco Chemie (Utrecht, The Netherlands). The equipment is driven by the general purpose electrochemical system (GPES) software version 4.9. A conventional three-electrode electrochemical cell system was used with Ag|AgCl (in 3 M KCl), platinum wire and platinum rod as the reference, counter and working electrodes, respectively.

### 3.5. Biological Activity

#### Antibacterial Study

The antibacterial activity of MHACD was studied against *Staphylococcus aureus* and *Enterococcus* species isolated from milk and groundwater samples in the North West Province, South Africa. The identities of the isolates were confirmed using standard preliminary and confirmatory microbiology tests. The isolates were obtained from the Molecular Microbiology Laboratory, Department of Biological Sciences, North-West University, Mafikeng Campus and used for the antimicrobial assay. Different concentrations of the ligand, namely 1 µg/mL, 2 µg/mL, 3 µg/mL and 4 µg/mL, were prepared with sterile distilled. Sterilized paper discs of uniform diameter (6 mm) were cut and sterilized by autoclaving. The paper discs were soaked in the standard solutions of the ligand for 10 min. Bacterial suspensions of *Staphylococcus aureus* and *Enterococci* were prepared and aliquots of 100 µL from each suspension were spread-plated on Muller Hinton agar. The paper discs were aseptically placed on inoculated plates and incubated at 37 °C for 24 h. Isolates were also tested against ligands while a disc with no ligand concentration was included in each inoculated plate as a negative control. The diameters of the zone of inhibition of discs were recorded for different concentrations of the ligand.

### 3.6. Corrosion Inhibition Study

#### 3.6.1. Metal Specimen and Inhibitor Solution

Mild steel (MS) specimens of the composition (wt %) 0.02 P, 0.37 Mn, 0.03 S, 0.01 Mo, 0.039 Ni, 0.21 C and balance Fe were cut into a square dimension of 1 cm × 1 cm and embedded in epoxy resin exposing a surface are of 1 cm^2^. Prior to each corrosion rate measurement, MS samples were abraded with different grades of emery papers (600 to 1200 grits), washed thoroughly with distilled water, degreased with acetone, rinsed with distilled water and finally air-dried.

The solution of the synthesized MHACD used as corrosion inhibitor was prepared in the concentration range of 10 ppm to 1000 ppm.

#### 3.6.2. Potentiodynamic Polarization Measurements

Electrochemical corrosion measurements of MS in 1 M HCl without and with various concentrations of the synthesized ligand as inhibitor were conducted using the potentiodynamic polarization method. The conventional three-electrode electrochemical cell comprising the MS with freshly polished surface as the working electrode (WE), Ag|AgCl, 3 M KCl as the reference electrode (RE) and platinum rod as the counter electrode (CE) was used for all the measurements. The electrochemical cell was connected to the Metrohm Autolab PGSTAT 302N supplied by Eco Chemie (Utrecht, The Netherlands). The MS was immersed in the aggressive solution for 30 min to ensure a stable open circuit potential (OCP) before each electrochemical measurement. The potentiodynamic polarization study was carried out by sweeping the MS electrode potential between −800 and −200 mV at a scan rate of 1 mV·s^−1^. The linear Tafel segments of the anodic and cathodic polarization curves were extrapolated to the corrosion potential E_corr_ to obtain electrochemical kinetic parameters including the corrosion current density (*i_corr_*), anodic (*β_a_*) and cathodic (*β_c_*) Tafel slopes. The percentage inhibition efficiency was calculated by using the equation:

(5) $$\%IE_{PDP}=\left(\frac{i_{corr}^{0}-i_{corr}}{i_{corr}^{0}}\right)\times 100$$

where $i_{corr}^{0}$ and $i_{corr}$ are corrosion current densities in the absence and presence of inhibitors, respectively.

The electrochemical corrosion measurements were conducted under unstirred conditions at 303 K.

#### 3.6.3. Quantum Chemical Study

Quantum chemical calculations were carried out to gain further insight into the correlation between the molecular structure of the synthesized ligand and its corrosion inhibition properties. The structure of MHACD was modeled with the GaussView 5.0 software to obtain the starting geometry after which geometry optimization was carried out using the Windows based Gaussian 09 suite software (version D.01) [55]. Full geometry optimization of MHACD was carried out without symmetry constraint using the B3LYP/6-31+G(d,p) model of density functional theory (DFT) comprising the Becke 3-Parameter exchange functional together with the Lee–Yang–Parr correlation functional (B3LYP) [56,57] used in combination with the 6-31+G(d,p) basis set. The frontier molecular orbital (FMO) energy parameters of the optimized structure of L including the energy of the highest occupied molecular orbital (E_HOMO_) and the energy of the lowest unoccupied molecular orbital (E_LUMO_) were calculated. The global electronegativity, χ (χ = −½(E_HOMO_ + E_LUMO_)) and hardness, η (η = −½(E_LUMO_ − E_HOMO_)) were also calculated. The fraction of electrons transferred (∆N) from the inhibitor molecule (donor) to the metallic (Fe) atom (acceptor) was calculated using the equation: [39,58].

(6) $$\Delta N=\frac{\chi_{Fe}-\chi_{inh}}{2(\eta_{Fe}+\eta_{inh})}$$

where *χ* and *η* denote the electronegativity and hardness, respectively. A value of 7 eV/mol was used for $\chi_{Fe}$, while $\eta_{Fe}$ was equated to 0 eV/mol for bulk Fe atom in accordance to Pearson’s electronegativity scale [59]. The natural bond orbital (NBO) analysis was also carried out to investigate the likely atomic orbitals of MHACD that are involved in donor–acceptor interactions with the Fe atomic orbitals during the adsorption and corrosion inhibition phenomenon.

## 4. Conclusions

The nickel(II) complex of 1,8-dimethyl-1,3,6,8,10,13-hexaazacyclotetradecane (NiMHACD) was synthesized and later demetallated to obtain the corresponding free macrocylic ligand MHACD. Both NiMHACD and MHACD were characterized using the FT-IR, ^1^HNMR, ^13^CNMR, UV-Vis, and EDX techniques. The free ligand, MHACD, was investigated for its antimicrobial activities, electrochemical redox activities and corrosion inhibition potentials. The following conclusions can be drawn from the results:

1) The results FT-IR, ^1^HNMR, ^13^CNMR, UV-Vis, and EDX characterization revealed successful synthesis of NiMHACD and dematallation to MHACD.
2) MHACD was found to exhibit anti-bacteria activities against *Staphylococcus aureus* and *Enterococcus* species, being more active against the latter and the zone of inhibition increases with increasing concentration of MHACD.
3) MHACD displayed electrochemical redox properties that suggest its possible catalytic properties in electrochemical applications.
4) Potentiodynamic polarization study suggested that MHACD is a mixed-type corrosion inhibitor for mild steel in 1 M HCl.
5) The adsorption of MHACD was found to be spontaneous, obey the Langmuir adsorption isotherm, and involve competitive physisorption and chemisorption mechanisms.
6) Quantum chemical study showed that the HOMO of MHACD is high enough to favor forward donation of charges to the metal, while various orbitals in the MHACD that are capable of donating or accepting electrons were identified using the NBO analysis.

## Figures and Tables

**Figure 1:** The UV-Vis absorption spectra of NiMHACD and MHACD.

**Figure 2:** Antibacterial activities of MHACD against *Staphylococcus aureus* and *Enterococcus* species as (**a**) zone of inhibition against *Enterococcus* species (A = 4; B = 1; C = 2; D = 3 µg/mL; and the control is the unlabeled white spot at the center of the disc); and (**b**) variation of inhibition diameter against concentration of MHACD.

**Figure 3:** Cyclic voltammograms for bare Pt electrode in 0.1 M PBS (pH 7.0) without and with 1 mM of MHACD at 25 mV·s^−1^ scan rate showing the relatively more: (**a**) cathodic potential region and (**b**) anodic potential region.

**Figure 4:** Effect of scan rate on the electrochemical behavior of MHACD at ν = 25–300 mV·s^−1^.

**Figure 5:** Plots of (**a**) log Ip *vs.* log ν and (**b**) E_p_ *vs.* log ν for MHACD.

**Figure 6:** Potentiodynamic polarization curves for MS in 1 M HCl without and with various concentrations of the inhibitor (MHACD).

**Figure 7:** Langmuir adsorption isotherm for MS in 1 M HCl containing various concentrations of MHACD at 303 K. The values of K_ads_ and ΔG_ads_ are listed on the graph.

**Figure 8:** Optimized structure (**a**); the highest occupied molecular orbital (HOMO) (**b**); and and lowest unoccupied molecular orbital (LUMO) (**c**) of MHACD. Only the non-hydrogen atoms are shown and numbered in the optimized structure such that: grey = Carbon; blue = Nitrogen. The numbering pattern in the optimized structure is used for discussion of the results.

**Figure 9:** Synthesis of (NiMHACD).

**Figure 10:** Demetallation of NiMHACD to obtain the metal-free ligand, MHACD.

**Table 1:** Fourier transform infra-red (FT-IR), proton nuclear magnetic resonance (^1^H-NMR), carbon-13 nuclear magnetic resonance (^13^C-NMR), ultraviolet-visible (UV-vis), and energy dispersive X-ray (EDX) spectroscopic data for the synthesized NiMHACD and MHACD.

NiMHACD	
FT-IR (v/cm^−1^)	1026s (C–N); 1503m (N–H, bend); 3222m (C–H, stretch), 3550b (N–H, stretch)
^13^C-NMR (CDCl_3_, δ, ppm)	39.90 (–N–CH_3_), 71.20 (–N–C–N–), 172.60 (–N–CH_2_–CH_2_–N)
^1^H-NMR (CDCl_3_, δ, ppm)	0.9 (s, 6H, –N–CH_3_), 1.2 (m, 8H, –N-CH_2_-CH_2_–N–), 1.5 (d, 8H, –N–CH_2_–N–), 7.2 (m, 4H, –C–NH–C–)
UV-vis (nm)	214 (^1^A_1g_ → ^1^A_2g_), 324 nm (^1^A_1g_ → ^1^B_1g_)
EDX	22.5% Ni
**MHACD**	
FT-IR (v/cm^−1^)	1421s (C–N); 1584m (N–H, bend); 3300b (N–H, stretch)
^13^C-NMR (CDCl_3_, δ, ppm )	28.56 (–N–CH_3_), 78.43 (–N–C–N–), 174.60 (–N–CH_2_–CH_2_–N)
^1^H-NMR (CDCl_3_, δ, ppm)	0.9 (s, 6H, –N–CH_3_), 1.3 (m, 8H, –N–CH_2_–CH_2_–N–), 1.6 (d, 8H, –N–CH_2_–N–), 7.3 (m, 4H, –C–NH–C–)
UV-vis (nm)	286 (n → σ*)
EDX	0% Ni

**Table 2:** Tafel parameters for MS corrosion in 1 M HCl without and with various concentrations of the inhibitor (L).

Inhibitor Conc. (ppm)	−*E*_corr_ (mV)	*i*_corr_ (mA·cm^−2^)	*b*_a_ (mV·dec^−1^)	*b*_c_ (mV·dec^−1^)	*%IE*_PDP_
–	–	Blank (1 M HCl)	–	–	–
–	467	2.838	134	185	–
–	–	Inhibitor (MHACD)	–	–	–
10	498	2.288	153	215	76.54
100	465	1.947	128	176	79.53
400	445	1.296	90	120	89.61
500	436	1.251	90	118	95.28
1000	464	0.581	86	129	98.58

**Table 3:** Selected bond lengths in the optimized structure of MHACD.

Geometry Parameter	Gas Phase
C1–N5	1.458
C6–N5	1.466
C6–N12	1.455
C9–N5	1.465
C9–N14	1.449
C16–N12	1.456
C19–N14	1.465
C16–C22	1.533
C19–C25	1.530
C22–N28	1.452
C25–N30	1.462
C32–N28	1.446
C35–N30	1.455
C32–N38	1.460
C35–N38	1.476
C39–N38	1.458

**Table 4:** Some quantum chemical parameters of the synthesized ligand (MHACD).

Quantum Chemical Parameters						
E_HOMO_ (eV)	E_LUMO_ (eV)	∆E (eV)	χ (eV)	η (eV)	∆N	Dipole Moment (Debye)
−4.17	0.11	4.27	2.03	2.14	1.16	1.74

**Table 5:** **Natural bond orbital (**NBO) analysis of the N atoms in the molecule of MHACD.

Atom	Orbital Type	Occupancy	Energy (a.u)
N5	2s	1.283	−0.517
	2px	1.576	−0.203
	2py	1.26	−0.187
	2pz	1.435	−0.195
N12	2s	1.339	−0.523
	2px	1.365	−0.179
	2py	1.639	−0.193
	2pz	1.35	−0.177
N14	2s	1.334	−0.525
	2px	1.249	−0.171
	2py	1.543	−0.189
	2pz	1.575	−0.197
N28	2s	1.333	−0.521
	2px	1.285	−0.174
	2py	1.502	−0.188
	2pz	1.59	−0.193
N30	2s	1.32	−0.514
	2px	1.265	−0.168
	2py	1.563	−0.184
	2pz	1.561	−0.188
N38	2s	1.291	−0.513
	2px	1.263	−0.182
	2py	1.256	−0.181
	2pz	1.728	−0.204

**Table 6:** Rydberg orbitals of C and N atoms in the molecule of MHACD.

Atom	Orbital Type	Energy (a.u)
C1	3dxy	2.164
C6	3dxz	2.206
C9	3dxy	2.180
C16	3dxz	2.133
C19	3dz^2^	2.077
C25	3dz^2^	2.092
C35	3dx^2^ − y^2^	2.209
C39	3dxz	2.239
N5	3dxy	2.122
N12	3dxy	2.190
N14	3dz^2^	2.103
N28	3dxz	2.179
N30	3dz^2^	2.098
N38	3dxz	2.094
